The article "Efficacy of Laparoscopic Radical Resection Combined with Neoadjuvant Chemotherapy and Its Impact on Long-Term Prognosis of Patients with Colorectal Cancer" was retracted in 2023. Reasons: signs of a paper mill; compromised peer review; unreliable results or conclusions.

# Efficacy of Laparoscopic Radical Resection Combined with Neoadjuvant Chemotherapy and Its Impact on Long-Term Prognosis of Patients with Colorectal Cancer

**DOI:** 10.1155/2022/4774531

**Published:** 2022-08-09

**Authors:** Liang Huang, Xijuan Xu, Jinfan Shao, Weiwen Hong, Wenfeng Yu

**Affiliations:** Department of Anus and Intestine Surgery, Taizhou First People's Hospital, Taizhou 318020, China

## Abstract

**Objective:**

The aim of the study is to examine the efficacy of laparoscopic radical resection of colorectal cancer combined with neoadjuvant chemotherapy and its impact on the overall prognosis of patients with colorectal cancer (CC).

**Methods:**

A total of 80 CC patients hospitalized and treated at our hospital between November 2019 and June 2021 were selected at random as research subjects and divided equally into two groups: the surgical group (*n* = 40) and the combination group (*n* = 40). Patients in the surgical group were treated with laparoscopic radical resection, while patients in the combination group received laparoscopic radical resection combined with neoadjuvant chemotherapy. The two groups were compared in terms of surgery-related indicators, tumor markers (serum carcinoembryonic antigen (CEA), glycoprotein 199 (CA199), vascular endothelial growth factor (VEGF), and matrix metalloproteinase 9 (MMP9)), postoperative complications, and 1–3 years postoperative survival rate and recurrence rate.

**Results:**

The surgical duration of the combination group was significantly shorter than the surgical group (*P* < 0.05). No significant differences were found in intraoperative blood loss, time to get out of bed, exhaust time, or hospital stay between the two groups (*P* < 0.05). In the combination group, serum tumor markers (carcinoembryonic antigen (CEA), carbohydrate antigen 199 (CA199), vascular endothelial growth factor (VEGF), and matrix metalloproteinase 9 (MMP9)) were markedly lower than those in the surgical group (*P* < 0.05). The combination group exhibited fewer postoperative complications than those in the operation group (*P* < 0.05). In the combination group, the 1–3 years postoperative survival rate was higher, while the 1–3 years postoperative recurrence rate was considerably lower than that in the surgical group (*P* < 0.05).

**Conclusion:**

CC patients benefit well from laparoscopic radical resection coupled with neoadjuvant chemotherapy. The approach is efficient in lowering blood tumor markers in patients and lowering the risk of surgery-related complications. It has the potential to enhance patients' long-term prognoses, allowing them to live longer and lower their chance of recurrence.

## 1. Introduction

Colorectal cancer (CC) is a common malignant tumor disease of the gastrointestinal tract, which mostly occurs in middle-aged females [1]. Incidence of the disease has been trending towards younger ages [2]. CC does not always exhibit obvious symptoms (involving hematochezia, diarrhea, constipation, and localized abdominal pain) in its early stage, while the disease progresses to advanced stages with systemic symptoms such as anaemia and weight loss [3]. CC is characterized by a high mortality rate. According to clinically related statistical studies, CC is second only to gastric cancer and esophageal cancer among digestive system malignant tumors in terms of the incidence and mortality [4]. Currently, the surgery is the mainstay of clinical treatment for CC. Besides, radiotherapy, chemotherapy, and targeted therapy are on the list of major interventions, among which chemotherapy offers definite efficacy on tumors, yet with more adverse reactions, including nausea, vomiting, diarrhoea, oral mucositis, and neurotoxicity, which limit its clinical application and reduce the quality of life of CC patients [5]. Therefore, it is a medical challenge to find safe and effective drugs to alleviate the adverse effects of chemotherapy, improve the immunity of patients, and avoid recurrence and metastasis rates after surgery [6]. Chinese medicine is highly effective against tumors which can effectively prolong the survival of patients, improve their quality of life, and reduce the adverse effects of chemotherapy [7]. According to traditional Chinese medicine, the main pathogenesis of colorectal cancer is phlegm and blood stasis, qi stagnation, qi and blood weakness, spleen and stomach weakness, spleen dysfunction, endogenous phlegm, blocked blood circulation, vein stasis, qi stagnation, and blood stasis. When phlegm and blood compete with each other and coagulate in the intestinal tract, cancer will occur.

The article "Efficacy of Laparoscopic Radical Resection Combined with Neoadjuvant Chemotherapy and Its Impact on Long-Term Prognosis of Patients with Colorectal Cancer" was retracted in 2023. Reasons: signs of a paper mill; compromised peer review; unreliable results or conclusions.

In recent years, the clinical curative rate among colorectal cancer patients has considerably improved on account of the development and advancement of medical technology and medical equipment in China. Despite this, Ma Xin have demonstrated that, while surgical therapy has a considerable clinical impact on colorectal cancer patients, the long-term prognosis for the majority of patients remains dismal [8]. CC patients are commonly treated with perioperative adjuvant therapy in the form of neoadjuvant chemotherapy, which can effectively reduce the tumor staging and progression grading of patients, which can further improve the curative rate and the long-term prognosis of patients [9]. The objective of this study was to investigate the efficacy of laparoscopic radical resection of colorectal cancer combined with neoadjuvant chemotherapy and its influence on long-term prognosis in 80 CC patients treated in our hospital. There is a reference to a clinical research study.

## 2. Materials and Methods

### 2.1. General Data

80 CC patients hospitalized and treated at our facility between November 2019 and June 2021 were chosen as research subjects randomly, and they were allocated into the surgical and combination group, with 40 cases in each group. The randomization was carried out using an online web-based randomization tool (freely available at http://www.randomizer.org/). For concealment of allocation, the randomization procedure and assignment were managed by an independent research assistant who was not involved in screening or evaluation of the participants. A total of 27 males and 13 females participated in the surgical group, ranging in age from 39 to 72, with an average age of (54.77 ± 8.96) years.

#### 2.1.1. Tumor Type

16 cases of colon cancer and 24 cases of rectal cancer were detected.

#### 2.1.2. Clinical Stage

11 cases of stage II, 21 cases of stage III, and 8 cases of stage IV were detected.

#### 2.1.3. Pathological Type

9 cases with high differentiation, 22 cases with moderate differentiation, and 9 cases with low differentiation were detected. In the combination group, there were 28 males and 12 females, aged 40–4 years, with an average age of (54.92 ± 8.89) years.

#### 2.1.4. Tumor Type

15 cases of colon cancer and 25 cases of rectal cancer were detected.

#### 2.1.5. Clinical Stage

13 cases of stage II, 19 cases of stage III, and 8 cases of stage IV were detected.

#### 2.1.6. Pathological Type

8 cases of high differentiation, 23 cases of moderate differentiation, and 9 cases of poor differentiation were detected.

Informed consent was obtained from patients and signed prior to enrolment in the study. The study protocol was approved by the hospital ethics committee. Ethics number: SHI-EW20190902. All processes were in accordance with the Declaration of Helsinki ethical guidelines for clinical research.

### 2.2. Inclusion and Exclusion Criteria

#### 2.2.1. Inclusion Criteria

The inclusion criteria were as follows:

- Those who were diagnosed with CC based on clinically relevant examination results
- Those who did not have any contraindications to surgery
- Those who and whose families were informed and volunteered to participate in this study

#### 2.2.2. Exclusion Criteria

The exclusion criteria were as follows:

- Those with psychiatric disorders
- Those who are unable to undergo surgery or are allergic to any of the drugs used in this study
- Those with poor compliance and who cannot cooperate effectively with the research team

The article "Efficacy of Laparoscopic Radical Resection Combined with Neoadjuvant Chemotherapy and Its Impact on Long-Term Prognosis of Patients with Colorectal Cancer" was retracted in 2023. Reasons: signs of a paper mill; compromised peer review; unreliable results or conclusions.

### 2.3. Methods

Patients in both the groups were given conventional treatment interventions on admission, which included interventions for the underlying disease and nutritional support for the patient's body.

- Patients in the surgical group underwent laparoscopic radical resection of colorectal cancer: the patients received general anesthesia with conventional tracheal intubation and CO_2_ pneumoperitoneum was established. An abdominal puncture of 10 millimeters, two punctures of 5 millimeters each in the left and right upper abdomen, and a laparoscope, which was used to view the intra-abdominal lesions. Based on the location and size of the patient's lesions, the patient underwent a radical colorectal resection. Dissociation of the colorectum, removal of regional lymph nodes, and stapler anastomosis were performed in the course of the operation. The patient's abdominal cavity was then flushed with irrigation fluid, and a silicone tube was routinely inserted for drainage. During the operation, the principle of no tumor should be strictly adhered to. Extracted tissue specimens were ligated by the specimen bag and removed from the small incision for pathological examination. The patients received adjuvant chemotherapy one month following surgery, for a total of 10 cycles of chemotherapy [8].
- The patients in the combination group received neoadjuvant chemotherapy based on the treatment given to the observation group: the combination group patients' reference standards and particular operation procedures were consistent with those of the surgery group patients. Before surgery, individuals in the combination group received three rounds of neoadjuvant chemotherapy (FOLFOX4 regimen). The treatment plan specifically included the following measures:

The patient received oxaliplatin injection on the 1st day (Jiangsu Hengrui Medicine Co., Ltd., approved by National Medicines Co., Ltd., H20000337), at a dose of 130 mg/m^2^ according to the body surface area, and for three to five hours; infusion of leucovorin calcium for 1 and 2 days (Chongqing Yaoyou Pharmaceutical Co., Ltd., Chinese medicine Zhunzi H2000615), the dosage is 200 mg/m^2^ based on the area of the body, continuous infusion for over 3 hours; intravenous infusion on the 1st and 2nd day 5-fluorouracil injection (Shanghai Xudong Haipu Pharmaceutical Co., Ltd., H31020593), the dose is 500 mg/m^2^ of body surface area, and it is administered intravenously through an infusion pump at a rate of 5 mL/h for 24 hours; adverse reactions that may occur during chemotherapy need to be closely monitored [10]. After three cycles of chemotherapy, a laparoscopic radical resection of colorectal cancer was performed.

The article "Efficacy of Laparoscopic Radical Resection Combined with Neoadjuvant Chemotherapy and Its Impact on Long-Term Prognosis of Patients with Colorectal Cancer" was retracted in 2023. Reasons: signs of a paper mill; compromised peer review; unreliable results or conclusions.

Both groups were treated with the Chinese herbal medicine *Angelica sinensis* blood tonic soup in this basis. The recipe is as follows: 12 g of *Angelica sinensis* and 60 g of *Astragalus membranaceus*. 200 ml of the decoction was boiled and divided into 2 doses in the morning and evening after meals. 1 dose was taken daily. Patients start taking it 5 d before surgery and take it until the 7th postoperative day.

### 2.4. Observation Indicators

The observation indicators were as follows:

1. Surgery-related indicators: The surgery-related indicators in this study were listed as follows: operation time, intraoperative blood loss, time to get out of bed, exhaustion, and hospital stay. These surgical indicators were recorded by our hospital's relevant medical staff.
2. Serum tumor markers: 5 ml of venous blood was drawn from the two groups of patients before and after surgery, and the supernatant was collected following centrifugation. ELISA was used to detect CEA and carbohydrates. The levels of CA199, VEGF, and MMP9 were determined strictly according to the instructions provided with the kit.
3. Postoperative complications: Postoperative complications may include infection of the incision, anastomotic bleeding, intestinal obstruction, and anastomotic leakage.
4. The 1–3-year postoperative survival rate and the recurrence rate: The relevant medical staff after the operation will conduct a three-year follow-up visit to the patients, a telephone follow-up every six months, and a door-to-door follow-up once every year. As part of the door-to-door follow-up, the relevant medical staff of our hospital recorded the 1–3-year postoperative survival rate and recurrence rate of patients.

### 2.5. Statistical Methods

SPSS 22.0 software was used for the data analysis. The measurement data were expressed as $\left(\bar{x}\pm s\right)$, and independent *t*-test samples were conducted and the enumeration data were expressed as the number of cases (%). The *χ*^2^ test was performed. *P* < 0.05 indicates a statistical significance.

## 3. Results

### 3.1. General Data

As for general data, there was no substantial difference between the two groups of patients (*P* < 0.05). See Table 1.

### 3.2. Comparison of Surgical Indicators

There were no significant differences in intraoperative blood loss, time spent getting out of bed, exhaust time, or hospital stay between the combination and surgical group (*P* < 0.05). See Table 2.

### 3.3. Evaluation of Serum Tumor Markers

Serum tumor markers CEA, CA199, VEGF, and matrix MMP9 were significantly decreased in the combination group after treatment compared to the surgical group before treatment (Table 3, *P* < 0.05).

The article "Efficacy of Laparoscopic Radical Resection Combined with Neoadjuvant Chemotherapy and Its Impact on Long-Term Prognosis of Patients with Colorectal Cancer" was retracted in 2023. Reasons: signs of a paper mill; compromised peer review; unreliable results or conclusions.

### 3.4. Comparison of Postoperative Complications

Postoperative complications were considerably fewer in the combination group than those in the surgical group. (*P* < 0.05). See Table 4.

### 3.5. Comparison of 1–3-Year Postoperative Survival Rate and Recurrence Rate

The 1–3-year postoperative survival rate was significantly higher in the combined group than in the surgical group (*P* < 0.05); the 1–3-year postoperative recurrence rate was significantly lower in the combined group than in the surgical group (*P* < 0.05). See Table 5.

## 4. Discussion

Colorectal cancer is a common malignant tumor disease of the gastrointestinal tract with a high mortality, recurrence and metastasis rate; therefore, its early detection and treatment is crucial [11]. According to epidemiological studies, colorectal cancer is the fourth most common malignancy among males and the third most common among females. In recent years, the incidence and death rate of colorectal cancer has been increasing in line with the work pressure and irregular diet of people. Surgical intervention is the favoured treatment for this disease, with laparoscopic radical colorectal cancer being the predominant option, offering effective inhibition of tumor progression and prolonged survival of patients [12]. However, surgery and anesthesia are stressors that can induce disruption of the intestinal barrier in patients, and intestinal flora is closely associated with the development of colorectal cancer [13]. According to scholars such as Li Jinjin, surgery alone cannot entirely eradicate cancer cells in the patient's body, resulting in a relatively high recurrence rate of the disease following surgery. [14]. Neoadjuvant chemotherapy is a systemic chemotherapy given to patients before laparoscopic surgery [15]. Clinical research has confirmed that preoperative neoadjuvant chemotherapy can reduce the tumor mass in the human body, as well as kill the tumors that cannot be observed with the naked eye. Wang Lan et al. [16] and others have demonstrated that the combination of these two treatments can effectively control the recurrence rate of the patients, which renders a good prognosis of the patients. Zhang Qi et al. [17] and other studies have informed us that neoadjuvant chemotherapy in patients before laparoscopic radical resection of colorectal cancer will result in significant intraoperative blood loss, which will adversely affect the field of vision during surgery, and thus, lead to increased rates of abdominal pain and other adverse conditions. Colorectal cancer, belonging to the category of “dirty poison,” “accumulation,” and “intestinal mushroom” in Chinese medicine, is located in the large intestine and related to the spleen and stomach. Patients with colorectal cancer are physically weak, the spleen and stomach fail to transport and transform, and the conduction function of the large intestine decreases, which leads to the accumulation of cancerous tumors due to internal stasis and toxins. In modern Chinese medicine, colorectal cancer is classified into 4 stages and 7 types of symptoms. In this study, *Angelica sinensis* is used to tonify the blood, invigorate the blood, remove phlegm, and eliminate blood stasis and Huangqi is used to tonify the spleen, benefit the qi, and nourish the blood source. In this recipe, *Astragalus membranaceus* is reused to give full play to its effect of tonifying spleen and lung qi, so as to breed the source of blood. Combined with *Angelica sinensis*, it has the effect of nourishing the blood. Yang-sheng causes yin to grow long, both blood and qi to flourish, and it has the effect of invigorating qi and generating blood.

The article "Efficacy of Laparoscopic Radical Resection Combined with Neoadjuvant Chemotherapy and Its Impact on Long-Term Prognosis of Patients with Colorectal Cancer" was retracted in 2023. Reasons: signs of a paper mill; compromised peer review; unreliable results or conclusions.

According to the results of this study, the operation time of the patients in the combination group was significantly less than that of the patients in the operation group; no significant differences were found in intraoperative blood loss, recovery time, and exhaust time. Collectively, the neoadjuvant chemotherapy will not affect intraoperative blood loss and other related indicators between the two groups. However, the operation time for the combination group was shorter than the surgical group, which may be due to the fact that the combination group received chemotherapy before surgery. Chemotherapy can induce tumor shrinkage in patients, thereby reducing the time required for surgery [18]. In recent years, the detection of serum tumor markers in CC patients carries considerable implications for the diagnosis, assessment of therapeutic efficacy, and prognostic outcome of oncological disease in clinic. CEA and CA199 are frequently used as clinical markers for the assessment of oncological disease, and their levels may be utilized to identify the tumor staging as well as the prognosis of the patients [19, 20]. In this study, the postoperative levels of CEA and CA199 were significantly lower in the combined group than in the surgical group, suggesting that preoperative neoadjuvant chemotherapy could be effective in improving the serum levels of CC patients, which in turn improved the prognosis of the patients. VEGF is a prerequisite for tumor growth and differentiation, and elevated levels of the protein will also contribute to angiogenesis in patients. MMP9 is known to breakdown extracellular matrix, allowing it to disrupt the basement membrane and matrix of nearby cells immediately close to the patient's body lesion, which increases tumor cell infiltration and exerts an undesirable influence on tumor progression and metastasis. [21]. MMP9 can also promote the expression of VEGF in the body, which further promotes the growth and spread of the tumor in the patient's body [22, 23]. According to the results of this study, the postoperative levels of VEGF and MMP9 in the combination group were significantly lower than those in the surgical group, indicating that neoadjuvant chemotherapy interventions could significantly inhibit the expression of VEGF, MMP9, and other cytokines, which could increase tumor growth in patients with reduced ability, resulting in further improvements in patients' outcome. The long-term prognosis of patients following laparoscopic radical resection of colorectal cancer is not ideal because the operation cannot eradicate all cancer-related factors in the body. The results of this study showed that the incidence of postoperative complications was much lower in the combination group than in the surgical group. Furthermore, the 1–3-year postoperative survival rate was considerably higher in the combination group than the surgical group. The 1–3-year postoperative recurrence rate in the combination group was much lower than in the surgical group, suggesting that preoperative neoadjuvant chemotherapy treatment can effectively minimize the frequency of surgical problems, increase long-term survival, and prevent cancer recurrence. A possible explanation may lie in the fact that neoadjuvant chemotherapy can help patients reduce the number of primary lesions, which in turn promotes the de-escalation and downstaging of colorectal cancer, thus improving the complete response rate of patients to treatment. Positive for this, patients are at reduced risk of postoperative complications and long-term disease recurrence [24, 25].

The article "Efficacy of Laparoscopic Radical Resection Combined with Neoadjuvant Chemotherapy and Its Impact on Long-Term Prognosis of Patients with Colorectal Cancer" was retracted in 2023. Reasons: signs of a paper mill; compromised peer review; unreliable results or conclusions.

However, the following issues stand out: small sample size, short observation period, and no long-term follow-up. It is expected that in future, more investigators could cooperate with patients to conduct clinical studies with larger samples, thus providing more clinical evidences for the research and application of such a method.

In conclusion, laparoscopic colorectal cancer radical resection coupled with neoadjuvant chemotherapy has a considerable effect on CC patients. The approach is known to lessen the probability of postoperative problems in addition to lowering the level of blood tumor markers in patients. This approach has a beneficial influence on patients' long-term prognosis, enhancing long-term survival rates, and lowering the likelihood of illness recurrence.

## Figures and Tables

**Table 1:** Comparison of general data between the groups $\left[\bar{x}\pm s,n\left(％\right)\right]$.

	Surgical group (*n* = 40)	Combination group (*n* = 40)	*t*/*x*^2^	*P*
*Gender*			0.058	0.809
Male	27	28		
Female	13	12		

Age (years)	39–72	40–74		

Average age (years)	54.77 ± 8.96	54.92 ± 8.89	-0.075	0.94

*Tumor type*			0.053	0.818
Colon cancer	16	15		
Rectal cancer	24	25		

*Clinical stage*			0.267	0.606
Stage II	11	13		
Stage III	21	19		
Stage IV	8	8		

*Pathological type*			0.081	0.776
Highly differentiated	9	8		
Moderately differentiated	22	23		
Poorly differentiated	9	9		

**Table 2:** Comparison of surgical indicators $\left(\bar{x}\pm s\right)$.

Item	Surgical group (*n* = 40)	Combination group (*n* = 40)	*t*	*P*
Surgical duration (min)	144.62 ± 40.26	125.28 ± 35.85	2.269	0.026
Intraoperative blood loss (mL)	102.29 ± 30.76	104.61 ± 29.54	−0.344	0.732
Time to get out of bed (d)	2.46 ± 0.53	2.57 ± 0.49	−0.964	0.338
Exhaust time (d)	2.77 ± 0.62	2.74 ± 0.70	0.203	0.84
Hospital stay (d)	11.58 ± 3.24	12.19 ± 3.37	−0.825	0.412

**Table 3:** Evaluation of serum tumor markers $\left(\bar{x}\pm s\right)$.

Item	Time	Surgical group (*n* = 40)	Combination group (*n* = 40)	*t*	*P*
CEA (ng/ml)	Preoperation	28.47 ± 7.36	29.48 ± 8.26	−0.577	0.566
	Postoperation	14.55 ± 4.14	8.87 ± 2.11	7.731	<0.001

CA199 (kU/L)	Preoperation	48.28 ± 14.29	50.45 ± 15.23	−0.657	0.513
	Postoperation	33.41 ± 9.58	19.66 ± 6.32	7.61	<0.001

VEGF (ng/L)	Preoperation	660.27 ± 143.52	657.35 ± 138.87	0.092	0.927
	Postoperation	509.67 ± 95.28	442.89 ± 84.53	3.316	0.001

MMP9 (ng/L)	Preoperation	568.74 ± 164.62	580.74 ± 156.11	−0.335	0.739
	Postoperation	411.53 ± 85.39	348.96 ± 78.44	3.413	0.001

**Table 4:** Comparison of postoperative complications [*n*(%)].

t	Surgical group (*n* = 40)	Combination group (*n* = 40)	*x * ^*2*^	*P*
Wound infection	4	1		
Anastomic bleeding	2	1		
Intestinal obstruction	2	0		
Anastomic leakage	2	1		
Overall incidence (%)	10 (25%)	3 (8%)	4.501	0.034

**Table 5:** Comparison of 1–3-year postoperative survival and recurrence rate [*n* (%)].

	Surgical group (*n* = 40)	Combination group (*n* = 40)	x^2^	*P*
*Survival rate (%)*				
1 year	32 (80%)	39 (98%)	16.547	<0.001
2 years	27 (68%)	34 (85%)	8.038	0.005
3 years	21 (53%)	30 (75%)	10.503	0.001

*Recurrence rate (%)*				
1 year	2 (5%)	0 (0%)	5.128	0.024
2 years	5 (13%)	1 (3%)	6.793	0.009
3 years	9 (23%)	3 (8%)	8.589	0.003

## Data Availability

All data generated or analysed during this study are included in this published article.
